The article "Effects of Early Nursing Monitoring on Pregnancy Outcomes of Pregnant Women with Gestational Diabetes Mellitus under Internet of Things" was published in 2022. Journal: Comput Math Methods Med.

# Effects of Early Nursing Monitoring on Pregnancy Outcomes of Pregnant Women with Gestational Diabetes Mellitus under Internet of Things

**DOI:** 10.1155/2022/8535714

**Published:** 2022-06-01

**Authors:** Linlin Lu, Tinglan Huang

**Affiliations:** Department of Obstetrics, Chenzhou No.1 People's Hospital, Chenzhou, 423000 Hunan, China

## Abstract

To analyze the effect of early nursing intervention based on fetal heart signal extraction algorithm and Internet of Things (IoT) wireless communication technology on the adverse pregnancy outcomes of pregnant women with gestational diabetes mellitus (GDM) and newborns, 88 pregnant women diagnosed with GDM who underwent the 75 g glucose tolerance test at 24-28 gestational weeks in the hospital were selected as the research objects. According to the different intervention methods, the patients were divided into 44 cases of the experimental group (nursing intervention based on maternal and infant monitoring system) and 44 cases of the control group (outpatient follow-up intervention). The results showed that the compliance score and diet compliance rate of patients in the experimental group were signally higher than those in the control group at 1 and 3 months after intervention (*P* < 0.05). The levels of fasting blood glucose (FBG), blood glucose 2 hours after the meal, and hemoglobin A1c (HbA1c) in the experimental group were lower than those in the control group at 1 and 3 months after intervention (*P* < 0.05). The number of giant babies, hypoglycemia, hyperbilirubinemia, fetal distress, premature delivery, and birth weight in the experimental group was all lower than those in the control group, while the Apgar scores were higher than that in the control group (*P* < 0.05). To sum up, the intervention based on the intelligent maternal and infant monitoring system could timely help pregnant women adjust their diet structure and optimize the management of blood glucose and blood lipids, thus effectively improving the adverse pregnancy outcome and maintaining the health of pregnant women and newborns.

## 1. Introduction

Gestational diabetes mellitus (GDM) mainly refers to diabetes that does not exist before pregnancy but appears after pregnancy, which is caused by abnormal glucose metabolism due to a series of physiological changes during pregnancy [1, 2]. Nowadays, with the improvement of people's living standards and the development of medical technology, the incidence of GDM is getting higher and higher [3]. If GDM is not treated in time, it is very detrimental to the health of pregnant women and fetuses [4–6]. For pregnant women, GDM can increase the mother's possibility of developing high blood glucose, high blood pressure, and preeclampsia. For the fetus, it can increase the incidence of abortion, intrauterine growth retardation (IUGR), fetal malformation, giant babies, neonatal distress syndrome, and neonatal hypercholesterolemia [7, 8]. Besides, the long-term effect of GDM on mothers and infants cannot be ignored, which can lead to an increased risk of diabetes and other chronic diseases in the future [9]. Therefore, it is necessary to perform the targeted nursing intervention for pregnant women and fetuses in the early stage of pregnancy.

The article "Effects of Early Nursing Monitoring on Pregnancy Outcomes of Pregnant Women with Gestational Diabetes Mellitus under Internet of Things" was published in 2022. Journal: Comput Math Methods Med.

Fetal heart rate (FHR) monitoring is an important way of prenatal examination. Through 20 minutes of FHR monitoring, the trend of FHR can be figured out intuitively from the fetal heart curve, whether the fetus intrauterine hypoxia can be judged, and fetal health status can be assessed, which is usually suitable for the fetus in the perinatal period [10, 11]. If the pregnant woman is at high risk with advanced age, or she has pregnancy complications, the FHR monitoring needs to be performed in advance to avoid that fetal hypoxia is not noticed in time [12]. Traditional fetal monitoring can only be performed in the hospital, so pregnant women require to run back and forth for prenatal examination, which brings great trouble to pregnant women. Moreover, the traditional cable is adopted for data signal transmission, with great technical limitations [13, 14]. The Internet of Things (IoT) is an extended and expanded network based on the Internet. Through sensing devices, any item can be connected to the Internet according to the agreed protocol for information exchange and communication to realize the intelligent identification, positioning, tracking, monitoring, and management of items [15]. In recent years, with the pervasiveness of IoT technology and wireless network technology, there are various kinds of portable monitoring equipment that shows the good effect, and they can effectively get rid of the limitations of traditional cable and assist the hospital to better monitor the vital signs of maternal and infant [16, 17]. Besides, in the past, the obtained fetal heart signals could only be analyzed according to the personal experience of physicians, and special fetal heart rate changes could not be identified. Hence, the artificial intelligence (AI) fetal heart signal processing algorithm was introduced to further improve the effectiveness of maternal and infant monitoring [18].

To sum up, the adoption of the combination of AI algorithm, IoT technology, and wireless network technology in maternal and infant monitoring is a hot topic for scholars. An intelligent maternal and infant monitoring system based on fetal heart signal extraction algorithm and IoT wireless communication technology was proposed and applied in the early nursing intervention of pregnant women diagnosed with GDM who received the 75 g glucose tolerance test at 24-28 gestational weeks. The influence of early nursing intervention based on fetal heart signal extraction algorithm and IoT wireless communication technology on adverse pregnancy outcomes of pregnant women with GDM and neonates was deeply discussed, to provide help for early clinical nursing monitoring of pregnant women with gestational diabetes.

The article "Effects of Early Nursing Monitoring on Pregnancy Outcomes of Pregnant Women with Gestational Diabetes Mellitus under Internet of Things" was published in 2022. Journal: Comput Math Methods Med.

## 2. Materials and Methods

### 2.1. The Research Objects

In this study, 88 pregnant women who were diagnosed with GDM by the 75 g glucose tolerance test at 24-28 gestational weeks in the hospital from October 10, 2018, to May 1, 2020, were selected as the research objects, and the age ranged from 20 to 38 years old. All patients and their family members understood and signed informed consent. This study had been approved by the ethics committee of the hospital.

The inclusion criteria were as follows: (I) patients who did not have diabetes before pregnancy, (II) patients who did not receive the systematic diabetes health education, (III) patients with complete clinical data, and (IV) patients with the biochemical parameters of regular follow-up visits.

The exclusion criteria were as follows: (I) patients who dropped out of the experiment, (II) patients with other metabolic diseases, (III) patients with hyperthyroidism, (IV) patients with mental diseases, (V) patients who were unwilling to cooperate with follow-up visits, and (VI) patients who previously took any medication that affected the glycolipid metabolism in pregnant women.

### 2.2. Grouping

Patients were randomly divided into experimental group (*n* = 44) and control group (*n* = 44). Patients in the experimental group received the intervention based on the intelligent maternal and infant monitoring system. Patients in the control group received the outpatient follow-up intervention.

For the outpatient follow-up intervention, exercise training and diet plan guidance were implemented face-to-face, and the traditional oral education on GDM was also given simultaneously.

For the intervention based on the intelligent maternal and infant monitoring system, the maternal and infant monitoring system was used to collect and organize maternal and infant physiological information and surrounding environment information. The real-time data were checked by the physicians on the mobile devices, and the maternal and infant status assessment was made based on the analysis results of the computer. Then, through WeChat and QQ, patients were given the targeted diet plan and exercise rehabilitation program. Furthermore, the information about GDM was sent to pregnant women every week. Patients were encouraged to eat at home as much as possible and use a glucose meter to measure blood glucose by themselves.

The article "Effects of Early Nursing Monitoring on Pregnancy Outcomes of Pregnant Women with Gestational Diabetes Mellitus under Internet of Things" was published in 2022. Journal: Comput Math Methods Med.

### 2.3. Fetal Heart Signal Extraction Algorithm

Most of the existing portable fetal heart signal acquisition equipment relied on battery power, with the problems of small storage space and limited energy. Hence, the median filtering algorithm was introduced and optimized accordingly. Median filtering [19] is a nonlinear digital filter technology that is often used to remove the impurities in images or other signals. In Equation (1), median filtering was used to get the midvalue of the sample set in the window scope.

(1) $$\begin{array}{c} H\left(m\right)=\text{median}\left[x\left(m-M\right)x\left(m-M+1\right)\cdots x\left(m\right)\cdots x\left(m+M\right)\right]. \end{array}$$

In Equation (1), [*x*(*m* − *M*)*x*(*m* − *M* + 1) ⋯ *x*(*m*) ⋯ *x*(*m* + *M*)] represented the sample set, and median[] represented the midvalue of 2*m* + 1 samples.

The problem of the traditional median filtering algorithm lay in the heavy sorting workload of the window, so the idea of the binary search was introduced to construct and optimize the median filtering algorithm. This algorithm only needed to sort the window data when it was used for the first time, use the binary search method [20] to find the elements to be replaced, and insert new elements in the process of window movement. In the subsequent operation, it only needed to adjust the new elements to complete the correct sorting of the window data.  Figure 1 shows the specific process.

### 2.4. Design of Maternal and Child Monitoring System Based on Internet of Things Technology

An intelligent maternal and infant monitoring system was designed by using the AI algorithm and IoT wireless communication technology, which was classified into the maternal and infant monitoring equipment and the hospital monitoring center. The maternal and infant monitoring equipment (Figure 2) was mainly used to collect the physiological parameters and surrounding environment conditions of pregnant women and fetuses and transmit the information to the hospital monitoring center. This equipment included the information collection sensor and the local wireless monitoring terminal. The information collection sensor used a miniature wireless fetal heart sensor and a miniature wireless uterine pressure sensor. The local wireless monitoring terminal was used for information sorting, display, and transmission.  Figure 3 shows the procedure of information processing.

The article "Effects of Early Nursing Monitoring on Pregnancy Outcomes of Pregnant Women with Gestational Diabetes Mellitus under Internet of Things" was published in 2022. Journal: Comput Math Methods Med.

The hospital monitoring center was the most vital part of the whole system, which could provide physicians with accurate results of data analysis, including the client and the central server. The central server (Figure 4) was used to receive and store the collected physiological information and surrounding environment information of pregnant women. The client was mainly for the hospital physicians who could log in to the client on mobile devices, check the real-time displayed data, and make the diagnosis based on the analysis results of the computer.

### 2.5. Observation Indexes

General sociological data of pregnant women were recorded, including age, height, weight, gestational week, number of pregnancies, the educational level (primary school, junior high school, high school, college for professional training, and bachelor degree or above), family income (<3,000 yuan, 3,000-5,000 yuan, 5,000-10,000 yuan, 10,000-30,000 yuan, or >30,000 yuan), and medical form (provincial and municipal medical insurance, the new rural cooperative medical insurance, or self-funded medical insurance). The compliance scores and compliance rate of the diet standards of pregnant women before and after intervention were recorded. Biochemical indexes of pregnant women before and after intervention were recorded, such as fasting blood glucose (FBG), postprandial blood glucose (PBG), hemoglobin A1c (HbA1c) levels, red blood cell (RBC), and hemoglobin (HGB). The Apgar scores [20], weight, and complications of the fetus at birth were recorded. The adverse events were recorded during the follow-up visits, such as pregnancy-induced hypertension (PIH), premature rupture of membranes, oligohydramnios, polyhydramnios, anemia, threatened abortion, and preeclampsia.

### 2.6. Statistical Methods

SPSS 19.0 was employed for data statistics and analysis. Mean ± standard deviation ($\overset{¯}{x}\pm s$) was how measurement data were expressed, and percentage (%) was how count data were expressed. One-way analysis of variance was used for pairwise comparison. The difference was statistically significant with *P* < 0.05.

## 3. Results

### 3.1. Comparison of the General Sociological Data of Patients between Two Groups

In Figure 5, there were insignificant differences between the experimental group and the control group in age, height, weight, gestational week, number of pregnancies, the educational level (primary school, junior high school, high school, college for professional training, and bachelor degree or above), family income (<3,000 yuan, 3,000-5,000 yuan, 5,000-10,000 yuan, 10,000-30,000 yuan, or >30,000 yuan), and medical form (provincial and municipal medical insurance, the new rural cooperative medical insurance, or self-funded medical insurance) (*P* > 0.05).

The article "Effects of Early Nursing Monitoring on Pregnancy Outcomes of Pregnant Women with Gestational Diabetes Mellitus under Internet of Things" was published in 2022. Journal: Comput Math Methods Med.

### 3.2. Comparison of the Compliance and the Compliance Rate of the Diet Standards between the Two Groups before and after Intervention

In Figure 6, there were no statistically significant differences in the compliance score and the compliance rate of the diet standards between the experimental group and the control group before intervention (*P* > 0.05). The compliance score and the compliance rate of the diet standards of patients in the experimental group at 1 and 3 months after intervention were observably higher than those in the control group, with significant differences (*P* < 0.05).

### 3.3. Comparison of Biochemical Indexes between the Two Groups before and after Intervention

In Figure 7, there were no considerable differences in FBG, blood glucose 2 hours after the meal, HbA1c levels, RBC, and HGB between the two groups before the intervention (*P* > 0.05). The levels of FBG, blood glucose 2 hours after the meal, and HbA1c in the experimental group at 1 and 3 months after intervention were markedly lower than those in the control group (*P* < 0.05). There was no statistically considerable difference in RBC and HGB between the experimental group and the control group at 1 and 3 months after intervention (*P* > 0.05).

### 3.4. Comparison of Neonatal Status between the Two Groups

The number of giant babies, hypoglycemia, hyperbilirubinemia, fetal distress, and premature delivery in the experimental group was evidently lower than that in the control group (*P* < 0.05) (Figure 8(a)). The Apgar scores at birth in the experimental group were obviously higher than that in the control group (*P* < 0.05) (Figure 8(b)). The birth weight of newborns in the experimental group was signally lower than that in the control group (*P* < 0.05) (Figure 8(c)).

### 3.5. Comparison of the Adverse Events between the Two Groups

In Figure 9, there were 2 patients with PIH, 1 patient with premature rupture of membranes, 1 patient with oligohydramnios, 0 patients with polyhydramnios, 2 patients with anemia, 0 patients with threatened abortion, and 1 patient with preeclampsia in the experimental group. In the control group, there were 4 cases of PIH, 5 cases of premature rupture of membranes, 3 cases of oligohydramnios, 2 cases of polyhydramnios, 6 cases of anemia, 1 case of threatened abortion, and 4 cases of preeclampsia. The incidence of adverse events in the experimental group was manifestly lower than that in the control group (*P* < 0.05).

## 4. Discussion

GDM is a special type of diabetes and is a risk factor for adverse pregnancy outcomes. It not only negatively affects the pregnant woman and the fetus but also poses a potential threat to the future health of the pregnant woman and newborn. Consequently, it is necessary to find an effective method for the early intervention of pregnant women with GDM [21, 22]. An intelligent maternal and infant monitoring system based on the AI algorithm and IoT wireless communication technology was designed. Meanwhile, 88 pregnant women diagnosed with GDM who underwent the 75 g glucose tolerance test in the hospital at 24-28 gestational weeks were enrolled. According to the different intervention methods, they were classified into the experimental group (the intervention based on intelligent maternal and infant monitoring system) and the control group (the outpatient follow-up intervention). The general sociological data were firstly compared between the two groups. The results reflected that there were insignificant differences between the experimental group and the control group in age, height, weight, gestational week, the number of pregnancies, the educational level (primary school, junior high school, high school, college for professional training, and bachelor degree or above), family income (<3,000 yuan, 3,000-5,000 yuan, 5,000-10,000 yuan, 10,000-30,000 yuan, or >30,000 yuan), and medical form (provincial and municipal medical insurance, the new rural cooperative medical insurance, or self-funded medical insurance) (*P* > 0.05). It provided the basis for the following research. The compliance scores and the compliance rate of the diet standards of patients in the experimental group were signally higher than those in the control group at 1 and 3 months after the intervention (*P* < 0.05). With the improvement of people's living standards, the nutritional intake of pregnant women during pregnancy is adequate, but the collocation of diet is not often very reasonable, and it is prone to the problem of excess energy during pregnancy [23, 24]. Hence, the intervention based on the intelligent maternal and infant monitoring system could help pregnant women adjust their diet structure in time and ensure a good compliance rate of the diet standards, thereby improving the compliance of pregnant women.

The article "Effects of Early Nursing Monitoring on Pregnancy Outcomes of Pregnant Women with Gestational Diabetes Mellitus under Internet of Things" was published in 2022. Journal: Comput Math Methods Med.

Chen Y et al. [25] applied the combination of IoT and exercise-based individualized nursing intervention in the treatment of 139 patients with GDM. The results showed that the IoT combined with individualized exercise-based nursing intervention could effectively improve patients' blood glucose, insulin resistance, and psychological state, thus significantly improving their pregnancy outcome and mental state. The levels of FBG, blood glucose 2 hours after the meal, and HbA1c in the experimental group at 1 and 3 months after the intervention were markedly lower than those in the control group (*P* < 0.05), which indicated that the intervention based on intelligent maternal and infant monitoring system was helpful for patients with GDM to optimize the blood glucose management and adjust and control the blood lipid indexes. The incidence of adverse events in the experimental group was remarkably lower than that in the control group (*P* < 0.05), which demonstrated that the intervention based on the intelligent maternal and infant monitoring system helped effectively reduce the complications of pregnant women and improve their pregnancy outcomes. Moreover, the number of giant babies, hypoglycemia, hyperbilirubinemia, fetal distress, premature delivery, and birth weight in the experimental group was notably lower than those in the control group, while the Apgar scores were higher than that in the control group (*P* < 0.05). The abnormal changes in substance metabolism or structure-function during fetal growth and development were caused by adverse environmental effects, such as maternal high blood glucose in patients with GDM. These adverse effects were possible to persist after birth or even throughout life. Furthermore, the intervention based on the intelligent maternal and infant monitoring system could effectively improve the adverse pregnancy outcome and maintain the physical and mental health of pregnant women and newborns [26].

## 5. Conclusion

An intelligent maternal and infant monitoring system based on the AI algorithm and IoT wireless communication technology was designed. Simultaneously, 88 pregnant women diagnosed with GDM who underwent the 75 g glucose tolerance test in the hospital at 24-28 gestational weeks were included as the research objects. According to the different intervention methods, they were classified into the experimental group (the intervention based on intelligent maternal and infant monitoring system) and the control group (the outpatient follow-up intervention). The results showed that the intervention based on the intelligent maternal and infant monitoring system could timely help pregnant women adjust their diet structure, ensure a good compliance rate of the diet standards, optimize blood glucose and lipid management, and improve the compliance of pregnant women, thereby effectively improving the adverse pregnancy outcome and maintaining the physical and mental health of pregnant women and newborns. Nevertheless, the follow-up time of pregnant women and newborns in this experiment is only three months, and the long-term data is not collected. Follow-up studies will collect patient data from larger regions and different conditions to further analyze the feasibility of clinical application of the maternal and infant monitoring system in this research. In conclusion, this experiment provided a theoretical reference for the early nursing intervention of pregnant women with GDM.

The article "Effects of Early Nursing Monitoring on Pregnancy Outcomes of Pregnant Women with Gestational Diabetes Mellitus under Internet of Things" was published in 2022. Journal: Comput Math Methods Med.

## Figures and Tables

**Figure 1:** Process diagram of optimizing the median filtering algorithm.

**Figure 2:** The schematic diagram of the whole structure of the intelligent maternal and infant monitoring system.

**Figure 3:** Data management process of the local wireless monitoring terminal.

**Figure 4:** The schematic diagram of the function of the central server system.

**Figure 5:** Comparison of the general sociological data of patients between two groups. (a) Age, height, and weight. (b) Gestational weeks and the number of pregnancies. (c) Educational level. (d) Family income. (e) Medical form.

**Figure 6:** Comparison of the compliance and the compliance rate of the diet standards between the two groups. (a) The compliance score. (b) The compliance rate of the diet standards. 0-2: before the intervention, 1 month after the intervention, and 3 months after the intervention. ∗ meant that compared with the experimental group, *P* < 0.05.

**Figure 7:** Comparison of metabolic biochemical indexes between the two groups before and after the intervention. (a) Fasting blood glucose. (b) Blood glucose 2 hours after the meal. (c) Hemoglobin A1c levels. (d) Red blood cell. (e) Hemoglobin. 0-2: before the intervention, 1 month after the intervention, and 3 months after the intervention. ∗ meant that compared with the experimental group, *P* < 0.05.

**Figure 8:** Comparison of neonatal status between the two groups. (a) Complications. (b) The Apgar scores. (c) Weight. ∗ meant that compared with the experimental group, *P* < 0.05.

**Figure 9:** Comparison of the adverse events between the two groups. (b1–b7) Pregnancy-induced hypertension, premature rupture of membranes, oligohydramnios, polyhydramnios, anemia, threatened abortion, and preeclampsia. ∗ meant that compared with the experimental group, *P* < 0.05.

## Data Availability

The data used to support the findings of this study are available from the corresponding author upon request.

## References

[1] Vince K., Perković P., Matijević R. (2020). What is known and what remains unresolved regarding gestational diabetes mellitus (GDM). *Journal of Perinatal Medicine*.

[2] Simmons D. (2019). GDM and nutrition-answered and unanswered questions-there’s more work to do!. *Nutrients*.

[3] Khambule L., George J. A. (2019). The role of inflammation in the development of GDM and the use of markers of inflammation in GDM screening. *Advances in Experimental Medicine and Biology*.

The article "Effects of Early Nursing Monitoring on Pregnancy Outcomes of Pregnant Women with Gestational Diabetes Mellitus under Internet of Things" was published in 2022. Journal: Comput Math Methods Med.

[4] Mistry S. K., Das Gupta R., Alam S., Kaur K., Shamim A. A., Puthussery S. (2021). Gestational diabetes mellitus (GDM) and adverse pregnancy outcome in South Asia: a systematic review. *Endocrinol Diabetes Metab.*.

[5] Li X., Yu D., Wang Y. (2021). The intestinal dysbiosis of mothers with gestational diabetes mellitus (GDM) and its impact on the gut microbiota of their newborns. *Can J Infect Dis Med Microbiol.*.

[6] Li Y., Li D., Cheng X. (2021). The association between expression of lncRNAs in patients with GDM. *Endocrine Connections*.

[7] Boriboonhirunsarn D., Sunsaneevithayakul P., Pannin C., Wamuk T. (2021). Prevalence of early-onset GDM and associated risk factors in a university hospital in Thailand. *Journal of Obstetrics and Gynaecology*.

[8] Immanuel J., Simmons D. (2017). Screening and treatment for early-onset gestational diabetes mellitus: a systematic review and meta-analysis. *Current Diabetes Reports*.

[9] Loegl J., Nussbaumer E., Cvitic S., Huppertz B., Desoye G., Hiden U. (2017). GDM alters paracrine regulation of feto-placental angiogenesis via the trophoblast. *Laboratory Investigation*.

[10] Lewandowska M. (2021). Gestational diabetes mellitus (GDM) risk for declared family history of diabetes, in combination with BMI categories. *International Journal of Environmental Research and Public Health*.

[11] Mack L. R., Tomich P. G. (2017). Gestational diabetes: diagnosis, classification, and clinical care. *Obstetrics and Gynecology Clinics of North America*.

[12] Moradi F., Ghadiri-Anari A., Enjezab B. (2020). COVID-19 and self-care strategies for women with gestational diabetes mellitus. *Diabetes and Metabolic Syndrome: Clinical Research and Reviews*.

[13] Yew T. W., Chi C., Chan S. Y. (2021). A randomized controlled trial to evaluate the effects of a smartphone application-based lifestyle coaching program on gestational weight gain, glycemic control, and maternal and neonatal outcomes in women with gestational diabetes mellitus: the SMART-GDM study. *Diabetes Care*.

[14] Lv Z., Qiao L., Li J., Song H. (2021). Deep-learning-enabled security issues in the Internet of Things. *IEEE Internet of Things Journal*.

[15] Urbanová J., Brunerová L., Nunes M. A., Brož J. (2020). MODY diabetes and screening of gestational diabetes. *Ceská Gynekologie*.

[16] Zhou X., Li Y., Liang W. (2021). CNN-RNN based intelligent recommendation for online medical pre-diagnosis support. *IEEE/ACM Transactions on Computational Biology and Bioinformatics*.

[17] Chen X., Zhang Y., Chen H. (2021). Association of maternal folate and vitamin B12 in early pregnancy with gestational diabetes mellitus: a prospective cohort study. *Diabetes Care*.

The article "Effects of Early Nursing Monitoring on Pregnancy Outcomes of Pregnant Women with Gestational Diabetes Mellitus under Internet of Things" was published in 2022. Journal: Comput Math Methods Med.

[18] Yu Z., Amin S. U., Alhussein M., Lv Z. (2021). Research on disease prediction based on improved DeepFM and IoMT. *IEEE Access*.

[19] Tieu J., Shepherd E., Middleton P., Crowther C. A. (2017). Interconception care for women with a history of gestational diabetes for improving maternal and infant outcomes. *Cochrane Database of Systematic Reviews*.

[20] Cnattingius S., Johansson S., Razaz N. (2020). Apgar score and risk of neonatal death among preterm infants. *The New England Journal of Medicine*.

[21] Poblete J. A., Olmos P. (2021). Obesity and gestational diabetes in pregnant care and clinical practice. *Current Vascular Pharmacology*.

[22] Morampudi S., Balasubramanian G., Gowda A., Zomorodi B., Patil A. S. (2017). The challenges and recommendations for gestational diabetes mellitus care in India: a review. *Front Endocrinol (Lausanne).*.

[23] Shankar M., Chan C. S., Frayne S. M., Panelli D. M., Phibbs C. S., Shaw J. G. (2021). Postpartum transition of care: racial/ethnic gaps in veterans’ re-engagement in VA primary care after pregnancy. *Womens Health Issues*.

[24] Sparks J. R., Ghildayal N., Hivert M. F., Redman L. M. (2022). Lifestyle interventions in pregnancy targeting GDM prevention: looking ahead to precision medicine. *Diabetologia*.

[25] Chen Y., Qiu C., Chen J., Li L., Xu J., Sheng Z. (2021). Effect of the internet combined with exercise-based individualized nursing intervention in patients with gestational diabetes mellitus. *Diabetology and Metabolic Syndrome*.

[26] Mutabazi J. C., Enok Bonong P. R., Trottier H. (2021). Integrating gestational diabetes and type 2 diabetes care into primary health care: lessons from prevention of mother-to-child transmission of HIV in South Africa - a mixed methods study. *PLoS One*.

